The article "Infectious Offspring: How Birds Acquire and Transmit an Avian Polyomavirus in the Wild" was retracted in 2013. Reasons: unreliable data; unreliable results or conclusions; concerns about the data.

# Infectious Offspring: How Birds Acquire and Transmit an Avian Polyomavirus in the Wild

**DOI:** 10.1371/journal.pone.0001276

**Published:** 2007-12-05

**Authors:** Jaime Potti, Guillermo Blanco, Jesús Á. Lemus, David Canal

**Affiliations:** 1 Estación Biológica de Doñana, Consejo Superior de Investigaciones Científicas (CSIC), Department of Evolutionary Ecology, Pabellón del Perú, Sevilla, Spain; 2 Instituto de Investigación en Recursos Cinegéticos (IREC) Consejo Superior de Investigaciones Científicas (CSIC)-Universidad de Castilla-La Mancha (UCLM) - Junta de Comunidades de Castilla-La Mancha (JCCM), Ciudad Real, Spain; 3 Department of Evolutionary Ecology, Museo Nacional de Ciencias Naturales (CSIC), Madrid, Spain; University of Bristol, United Kingdom

## Abstract

Detailed patterns of primary virus acquisition and subsequent dispersal in wild vertebrate populations are virtually absent. We show that nestlings of a songbird acquire polyomavirus infections from larval blowflies, common nest ectoparasites of cavity-nesting birds, while breeding adults acquire and renew the same viral infections via cloacal shedding from their offspring. Infections by these DNA viruses, known potential pathogens producing disease in some bird species, therefore follow an ‘upwards vertical’ route of an environmental nature mimicking horizontal transmission within families, as evidenced by patterns of viral infection in adults and young of experimental, cross-fostered offspring. This previously undescribed route of viral transmission from ectoparasites to offspring to parent hosts may be a common mechanism of virus dispersal in many taxa that display parental care.

## Introduction

Arthropods are well-characterized vectors of many viruses of plants and animals [1], [2], including arboviruses (a non-systematic grouping of arthropod-borne, mostly RNA, viruses of vertebrates, where viral replication occurs in both the vertebrate and invertebrate hosts [3]). Although patterns of pathogen transmission are central to the evolution of infectious disease and host resistance [4]–[6], including those related to arboviruses [3], most of our knowledge stems from rather loose patterns of virus dispersal from broad, life-cycle perspectives which generally lack detailed information on the realized modes of virus dispersal across hosts at the population level [3]. The main modes of virus dispersal are vertical transmission, from a parent (usually the mother) to the offspring across host generations, and horizontal transmission, such as transmission through contact with infected non-parental individuals or objects in the environment. In a search for the effects that nest ectoparasitic blowflies (*Protocalliphora azurea* (Fallén)) may have on the biology of a forest passerine migrant species, the European pied flycatcher (*Ficedula hypoleuca* (Pallas)) [7], we screened birds' blood for the prevalence of several virus groups (including circovirus, polyomavirus, reovirus, smallpox and West Nile virus), and discovered a high degree of association between the presence of blowflies in the nest and polyomaviruses in the nestlings.

Polyomaviruses are a group of small, double-stranded DNA viruses best known from mammals and birds [8], though also present in lower vertebrates [9]. They have potential, confirmed pathogenic etiology and morbidity in at least man [10], apes, mice, parrots and finches, among a few other taxa [11]–[13]. Apart from horizontal virus transmission within flocks of caged parrots and other pet bird species there is no published information [8], [11] on how polyomavirus infections are primarily acquired *before* they jump across individual hosts.

The modes of polyomavirus acquisition in this study system are clearly limited by the known biology of its rather specialized, putative vector, as no larvae of Holarctic species of *Protocalliphora* have ever been recorded parasitizing individuals other than nestling birds. In pied flycatchers, eggs laid in the nest by the adult fly will hatch into larvae that develop to the pupal stage (our sampling unit) by hiding in the nest material. During this period, the larvae will take intermittent blood meals from nestlings, and will then burrow into the nest cup to pupate [14]. Blood-sucking by blowflies has a direct effect upon the nestlings, by rendering them anemic, decreasing their growth, and increasing their risk of mortality [14]–[17]; effects of the larvae on the parents are indirect, such as through causing them to increase their feeding rates to chicks [18]. This life-cycle immediately suggests a role for nestlings as the main agents of virus acquisition and eventual dispersal to the population as a whole. Alternative routes of virus dispersal may, however, complicate the pattern. For instance, vertical transmission from mothers to offspring via the egg, may also exist [19]. There is, furthermore, the possibility of horizontal transmission among related and unrelated individuals or objects in the environment (e.g., other nest parasites).

In this study, we evaluated whether the presence of an avian polyomavirus (APV hereafter) infecting nestlings of the pied flycatcher is associated with the presence of the nest ectoparasitic blowfly *P. azurea*, to assess its potential as vector of the virus. After dissecting the patterns of APV prevalence in adult and young birds in relation to ectoparasite prevalence, we performed an experiment to discard alternative routes of virus transmission across host generations.

## Results and Discussion

Prevalences of infection of APV in pied flycatcher blood were similarly high in nestlings in both study years (63.4%, *n* = 568 and 48.5%, *n* = 641 in 2005 and 2006, respectively) and breeding females (46.5%, *n* = 129 and 61.8%, *n* = 131, in 2005 and 2006, respectively; nestlings vs. females: χ^2^_1_ = 0.26, *P* = 0.61, pooling both years and applying Yates' correction for continuity) and lower in breeding males (37.1%, *n* = 116 and 39.7%, *n* = 121, in 2005 and 2006, respectively; males vs. females: χ^2^_1_ = 17.47, *P*<0.001; males vs. nestlings χ^2^_1_ = 22.95, *P*<0.001) while a sex difference in virus prevalence did not exist at fledging age (χ^2^_1_ = 0.03, *P* = 0.87, *n* = 184 male and 188 female nestlings from 2005 sexed with molecular methods [7]). Blowfly prevalence and APV presence in blood were tightly associated in both years, with all nests infested by blowflies containing at least one nestling infected by APV while only one brood out of 89 had a single nestling positive for APV in uninfested nests (Fisher's exact test, *P*<0.0001). The abundance scores of another nest ectoparasite (*Dermanyssus* Duges mites [7], [15]) were unrelated to the prevalence of APV in nestlings and adults (broods: χ^2^_1_ = 0.40, *P* = 0.53, females: χ^2^_1_ = 0.53, *P* = 0.47; males: χ^2^_1_ = 0.21, *P* = 0.65, pooling both years and applying Yates' correction for continuity) and all mites were negative for APV (*n* = 120).

The striking association found in both study years suggests that the transmission of the virus occurs from blowflies to offspring, and subsequently from offspring to parents, and not in the opposite direction, as virtually no nestlings from uninfested nests were infected with the virus (one out of 426 nestlings, Fig. 1) despite the infection of parents in many cases (Fig. 1). This discards possible transmission routes such as oral contact or aerosol spreading from infected parents to their nestlings. Furthermore, the likelihood that all nestlings in a brood were infected by APV increased with the number of blowfly larvae present in their nests. Only nestlings with six or less parasitic larvae in their nests could escape APV infection (Fig. 2). Adults, especially females, showed a similar association between APV infection and presence (Fig. 1) and abundance of blowflies in their nests (logistic regressions: 2005: females: *B* = 0.27, Wald = 22.79, *P*<0.0001, *n* = 123: males: *B* = 0.14, Wald = 12.95, *P*<0.0001, *n* = 109; 2006: females: *B* = 0.36, Wald = 14.68, *P*<0.0001, *n* = 116; males: *B* = 0.02, Wald = 0.40, *P* = 0.53, *n* = 96). Broods also resembled their parents, females in particular, as to prevalence of APV (Chi-square tests with Yates' correction for continuity; 2005: females: χ_1_^2^ = 6.22, *n* = 124, *P* = 0.013; males: χ_1_^2^ = 6.58, *n* = 113, *P* = 0.010; 2006: females: χ_1_^2^ = 7.84, *n* = 66, *P* = 0.005; males: χ_1_^2^ = 0.14, *n* = 59, *P* = 0.70).

**Figure 1:** Prevalence of APV infections in blood of nestlings and adult pied flycatchers in relation to presence or absence of nest ectoparasitic blowflies. 2005 nestlings: Fisher's exact test, *P*<0.0001; adult males: χ^2^_1_ = 6.00, *P* = 0.014; adult females: χ^2^_1_ = 5.99, *P* = 0.014; 2006 nestlings: χ^2^_1_ = 531.74, *P*<0.0001; adult males: χ^2^_1_ = 0.80, *P* = 0.370; adult females: χ^2^_1_ = 19.74, *P*<0.0001. The Yates' correction for continuity was applied. Numbers above bars are sample sizes (numbers of individuals).

**Figure 2:** Relationship between the number of blowflies in the nest and the prevalence of APV in nestlings in both study years. Logistic regressions; 2005: *B* = 1.05, Wald = 118.61, *P*<0.0001, *n* = 535; 2006: *B* = 2.55, Wald = 90.22, *P*<0.0001, *n* = 625.

The correspondence between the prevalences of blowflies and APV, on the one hand, and between APV infections in nestlings and their parents, on the other, points to genetic and/or environmental sources of resemblance between parents and offspring, e.g. in susceptibility or common exposure to APV infections, as potential sources of confusion in the interpretation of the routes of transmission of APV in this system. We therefore performed a cross-fostering experiment of whole clutches to test the hypotheses of parent-offspring similarity in patterns of APV infection due to vertical transmission of APV through the egg [19], or to genetic resistance to APV. The experiment showed that the APV status of infection in cross-fostered broods resembled that of their foster parents, females in particular (females: Fisher's exact test, *P* = 0.00003, *n* = 45; males: Fisher's exact test, *P* = 0.72, *n* = 35), rather than their genetic parents (females: χ_1_^2^ = 1.03, *n* = 38, *P* = 0.31; males: χ_1_^2^ = 0.88, *n* = 24, *P* = 0.88). This result indicates that APV is not passed to offspring from the mother, as occurs in mice [20], and discards the notion of strictly vertical (i.e. from parents to offspring) transmission of the virus.

Therefore, both natural patterns of infection in parents and offspring and experimental evidence with cross-fostered broods point to a common environmental primary source of infection, most likely the larvae of *P. azurea*. Analyses of 40 live blowfly larvae whose oral region was dissected and screened for APV presence supported the inferred pattern of virus transmission to nestlings, with 100% of foregut samples of the larvae exhibiting positive evidence for APV presence, most probably due to the likely installation of the virus in the salivary glands of its vector. APV was more rarely detected in the hindgut samples of the same blowfly individuals (15%, *n* = 40, of which 34 had empty guts and 6 had recently fed).

Our results point to the most plausible route of APV infection from nestlings to both their male and female parents as being through the parents' nest sanitation tasks. This is clearly supported by the finding that most APV-positive nestlings from nests infested by blowflies were actively shedding the virus in the sampled feces (85.0%, *n* = 40 nestlings from 26 nests) while APV was not isolated in feces from nestlings which had no detectable APV presence in blood (0%, *n* = 27 nestlings from 19 nests; Fisher's exact test, *P*<0.0001). This excludes the possibility of nestlings showing APV infection in the digestive tract with APV passing unnoticed in blood. Both sexes remove fecal sacs in the pied flycatcher but, as in other bird species [21], females are reported to do so at higher rates than males, in addition to swallowing them up to day three of nestling age [22]. Thus, both female-biased nest sanitation behavior and patterns of APV prevalence in feces support an APV vertical, ‘upwards’ route of transmission from offspring to parents, especially females. Also, a higher intensity of infection (as assessed by absolute quantification of viral gene copies [23]) in nestlings than in adults (Fig. 3) makes it more likely that nestlings were shedding the APV in feces [24], increasing the chance of transmission of APV to adults through their removal of fecal sacs.

**Figure 3:** Intensities of infection by APV in nestlings and adult birds. Shown are mean±SD scores quantifying the number of viral gene copies as assessed by RT-PCR Mann-Whitney U-tests give highly significant differences (*P*<0.001) for all possible between-group comparisons in both years. Numbers above bars are sample sizes (numbers of individuals).

To our knowledge, larvae of *P. azurea* are the first recorded vector for any polyomavirus, which may in turn be considered, under epidemiological criteria, both as an arbovirus [3] and an enteric virus (i.e., acquired through fecal-oral transmission [25]). African swine fever virus was the only previously known DNA-arbovirus [3], [11], a group to which APV of pied flycatchers should be added henceforth. As in tick arbovirus-vertebrate interactions [3], blowfly larvae surely inject APV through the wounds they produce with their sucking action into the bloodstream of nestling flycatchers during meals. This is consistent with the high intensity of infection displayed in the blood of nestlings, as compared to the reduced intensity of infection in adults (Fig. 3). However, lower intensities of infection in highly immunocompetent adults when compared to naïve, young individuals are also to be expected [3]. Furthermore, a low intensity of infection in adult birds may also reflect the fact that APV reaches adult individuals via a less direct route (through nestling feces) than the simple injection of viruses into the bloodstream by the parasite, as occurs in nestlings. In addition to the persistence of APV after infection in early life, which was confirmed one year later for all individuals already infected as nestlings (with only one exception, *n* = 13), brooding females could also be directly infected by attacks from blowfly larvae, as seemingly apparent from the increase in APV prevalence in females with the greater number of blowfly larvae counted in their nests. However, neither our long-term hands-on experience (23 years) with flycatchers nor the literature support the possibility that blowfly larvae ever attach to adult birds. Furthermore, excluding common infections as nestlings, a similar but weaker relationship in male flycatchers cannot be explained by the same mechanisms as in females, because males do not incubate or brood nestlings [22] and thus are unexposed to attacks by blowfly larvae. Therefore, common APV infections in adults and nestlings sharing a nest most likely reflect contagion from the nestling to the adult via cloacal shedding [26], with the virus jumping to parents as a result of their nest sanitation behavior, especially to females when swallowing feces. Intensity of infection in females could also be increased due to virus reactivation during breeding as occurs in mice during pregnancy [27], which necessitates further research.

The design and results of this study only allow us to speculate on where the APV infection originates, as all blowflies were positive for APV and the virus was only detectable in their primary (and, most probably, exclusive from the point of view of first transmission) host, the nestlings, when and *only* when their nest was infested by blowflies. However, this circle on the ‘true’ source of virus infection could be addressed at different levels of explanation. One hypothesis is that the non-parasitic, adult female flies may transmit the APV via vertical transmission through their eggs (transovarial transmission), and then throughout the larval (and pupal) stages to the adults (transstadial transmission) as known for some arboviruses [3]. This hypothesis, however, leaves unresolved the issue of the origin of infection by displacing the problem to the former fly generation. Studies of the biology of adult flies, e.g. of their food habits [14], could offer some clues on an earlier, ‘ultimate’ source of infection and also on whether all adult flies are reservoirs for APV. A complementary hypothesis, however, could make superfluous that search for the viral ‘origin’ by addressing the question of whether there has been joint cospeciation of APV of pied flycatchers and the blowfly *P. azurea*. We think this issue might be most profitably addressed through phylogenetic analysis of APV variants within the family Calliphoridae and, ideally, also within its sister group, flies in the family Sarcophagidae [28], [29].

In conclusion, nest ectoparasites of birds transmit polyomaviruses to nestlings, which in turn pass them on to their parents. To our knowledge, this is the first known natural example of a primary, rather than sporadic, route of upward transmission of a potential pathogen from offspring at an early ontogenetic stage to adult individuals. This route of infection may reveal itself as a common mechanism of virus transmission in the many taxa that exert parental care and/or feed and preen their offspring and thus might be a hitherto unnoticed [30] cost of parental care, with potential differences between the sexes depending on their roles in breeding tasks. Further, the arthropod to offspring to parent hosts route of virus transmission should probably be explored for other viral infections. Finally, given that pied flycatchers share breeding cavities and parasites with many other species [31], the findings reported here may open new research agendas on the evolution of virulence and cospeciation of vectors, virus and vertebrate hosts in the wild [3]–[6], [8], [32], [33], with added important potential implications of concern in conservation biology [34], [35].

## Materials and Methods

### Field methods

The study was conducted in 2005 and 2006 in an intensively studied population of pied flycatchers breeding in nest boxes in central Spain [7]. We recorded breeding phenology and reproductive success in all nests (*n* = 273) and trapped almost all breeding males and females within their nests while they fed nestlings aged 8–11 days. Nestlings were sampled at 13 days of age. A drop of blood was extracted from the brachial vein of all individuals and stored frozen in EDTA for molecular sex determination of nestlings [7] (only in 2005) and virological analyses (both years). Nest contents were removed after breeding and the nestboxes were cleaned again just before the breeding season. Thirty nestlings died in their nests before fledging, of which 12 were positive for APV and 18 negative.

### Cross-fostering experiment

In 2006, we exchanged all eggs in the second day of incubation between matched pairs of nests of the same (±1 d) breeding date and clutch size. Experimental nest dyads (*n = *94 nests, i.e. 47 dyads) were at least 1 km apart. Cross-fostered eggs were replaced by the same number of rubber, blue-painted canary egg dummies mimicking size and color of pied flycatcher eggs to avoid desertion by the females during clutch exchanges. In all cases, females ‘incubated’ the egg dummies during the time needed for transportation, as indicated by direct observation or our estimated temperature of egg dummies. Eggs were kept safe and warm in water-heated containers (cotton-coated, commercial hen egg packs) and transported by car in about 20 to 30 min. As a result of our procedure, all pairs of exchanged nests contained broods reared by totally unrelated adult birds. Final sample sizes were unbalanced due to some nests being lost to predation or because we were unable to trap the parent(s).

### Ectoparasite assessment

The abundance of blowflies was assessed by dismantling nest contents just after the young fledged and counting the number of pupae buried in the nest material. The abundance of mites, which can range from zero to thousands [15], was visually estimated as low or high on the day the fledglings were bled. These bimodal scores are highly predictive indices of the intensities of mite infestations, as shown by mite counts in Berlese funnels [15].

### Viral detection and quantification

Blood samples from adult and nestling pied flycatchers were tested for the presence of APV by means of a sensitive and specific real-time quantitative PCR (RQ-PCR) assay. Following previous work with a murine polyomavirus [23], the target sequences used for quantification of viral and cellular genes included the N termini of the T-antigens of APV (large, middle and small) and sequences of intron 3 within the avian wild-type p53 gene. P53 primers were used as a cellular normalization standard to allow calculations of viral genome copies per cell. Absolute quantification of viral gene copies was determined from standard curves generated by plotting the log_10_ of the known input gene copy number of the standard dilution series against the C_T_ value observed in the RQ-PCR analysis. Semi quantitative scores (from 1 to 5) were calculated by using 10 increment copies, so 0 is 0 copies detected, 1 from 10 to 10^2^ copies; 2 from 10^2^ to 10^3^ copies, 3 from 10^3^ to 10^4^ copies; 4 from 10^4^ to 10^5^ and, finally, 5 from 10^5^ to 10^6^ copies. Detection of APV in nestling feces, blow fly larvae and *Dermanyssus* mites was conducted by using a classical PCR assay [36]. A brood was defined as infected by APV when at least one nestling was positive for APV.

## References

[1] Gray SM, Banerjee N (1999). Mechanisms of arthropod transmission of plant and animal viruses.. Microbiol Mol Biol Rev.

[2] Carn VM (1996). The role of dipterous insects in the mechanical transmission of animal viruses.. Br Vet J.

[3] Kuno G, Chang G-JJ (2005). Biological transmission of arboviruses: reexamination of and new insights into components, mechanisms, and unique traits as well as their evolutionary trends.. Clin Microbiol Rev.

[4] Ewald PW (1994). Evolution of infectious disease..

[5] Levin BR (1996). The evolution and maintenance of virulence in microparasites.. Emerg Infect Dis.

[6] Lipsitch M, Siller S, Nowak MA (1996). The evolution of virulence in pathogens with vertical and horizontal transmission.. Evolution.

[7] Potti J, Dávila JA, Tella JL, Frías Ó, Villar S (2002). Gender and viability selection on morphology in fledgling pied flycatchers.. Mol Ecol.

[8] Pérez-Losada M, Christensen RG, McClellan DA, Adams BJ, Viscidi RP (2006). Comparing phylogenetic codivergence between polyomaviruses and their hosts.. J Virol.

[9] Essbauer S, Ahne W (2001). Viruses of lower vertebrates.. J Vet Med B.

[10] Lednicky JA, Butel JS (1999). Polyomaviruses and human tumors: a brief review of current concepts and interpretations.. Front Biosci.

[11] Villarreal LP (2006). Viruses and the evolution of life..

[12] Ritchie BW, Niagro FD, Latimer KS (1991). Polyomavirus infections in adult psittacine birds.. J Assoc Avian Vet.

[13] Johne R, Müller H (1998). Avian polyomavirus in wild birds: genome analysis of isolates from Falconiformes and Psittaciformes.. Arch Virol.

[14] Bennett GF, Whitworth TL (1991). Studies on the life history of some species of Protocalliphora (Diptera: Calliphoridae).. Can J Zool.

[15] Merino S, Potti J (1995). Mites and blowflies decrease growth and survival in nestling pied flycatchers.. Oikos.

[16] Hurtrez-Boussès S, Perret P, Renaud F, Blondel J (1997). High blowfly parasitic loads affect breeding success in a Mediterranean population of blue tits.. Oecologia.

[17] Hurtrez-Boussès S, Blondel J, Perret P, Renaud F (1997). Relationship between intensity of blowfly infestation and reproductive success in a Corsican population of blue tits.. J Avian Biol.

[18] Hurtrez-Boussès S, Blondel J, Perret P, Fabreguettes J, Renaud F (1998). Chick parasitism by blowflies affects feeding rates in a Mediterranean population of blue tits.. Ecol Lett.

[19] Mims CA (1981). Vertical transmission of viruses.. Microbiol Rev.

[20] McCance DJ, Mims CA (1977). Transplacental transmission of polyoma virus in mice.. Infect Immun.

[21] Hurd PL, Weatherhead PJ, McRae SB (1991). Parental consumption of nestling feces: good food or sound economics?. Behav Ecol.

[22] Cramp S, Perrins CM (1993). Handbook of the birds of Europe, the Middle East and North Africa volume VII: flycatchers to shrikes..

[23] Zhang S, McNees AL, Butel JS (2005). Quantification of vertical transmission of Murine polyoma virus by real-time quantitative PCR.. J Gen Virol.

[24] Phalen DM, Fudge AM (2000). Avian viral diagnostics.. Laboratory Medicine. Avian and Exotic pets.

[25] Murphy FA, Gibbs EPJ, Horzinek MC, Studdart MJ (1999). Veterinary virology, 3rd ed..

[26] Phalen DN, Radabaugh S, Dahlhausen RD, Styles DK (2000). Viremia, virus shedding, and antibody response during natural avian polyomavirus infection in parrots.. J Am Vet Med Assoc.

[27] McCance DJ, Mims CA (1979). Reactivation of polyoma virus in kidneys of persistently infected mice during pregnancy.. Infect Immun.

[28] Rognes K (1997). The Calliphoridae (Blowflies) (Diptera: Oestrioidea) are not a monophyletic group.. Cladistics.

[29] Stevens J, Wall R (2001). Genetic relationships between blowflies (Calliphoridae) of forensic importance.. Forensic Sci Int.

[30] Clutton-Brock TH (1991). The evolution of parental care..

[31] Lundberg A, Alatalo RV (1992). The pied flycatcher..

[32] Shadan FF, Villarreal LP (1996). The evolution of small DNA viruses of eukaryotes: past and present considerations.. Virus Genes.

[33] Villarreal LP, Defilippis VR, Gottlieb KA (2000). Acute and persistent viral life strategies and their relationship to emerging diseases.. Virol.

[34] Daszak P, Cunningham AA, Hyatt AD (2000). Emerging infectious diseases of wildlife - threats to biodiversity and human health.. Science.

[35] LaDeau SL, Kilpatrick AM, MarraLaDeau PP (2007). West Nile virus emergence and large-scale declines of North American bird populations.. Nature.

[36] Phalen DN, Wilson VG, Graham DL (1991). Polymerase chain reaction assay for avian polyomavirus.. J Clin Microbiol.

